The article "Age-Related Decline in Vertical Jumping Performance in Masters Track and Field Athletes: Concomitant Influence of Body Composition" was published in 2021. Journal: Front Physiol.

# Age-Related Decline in Vertical Jumping Performance in Masters Track and Field Athletes: Concomitant Influence of Body Composition

**DOI:** 10.3389/fphys.2021.643649

**Published:** 2021-04-01

**Authors:** José R. Alvero-Cruz, Mieszko Brikis, Phil Chilibeck, Petra Frings-Meuthen, Jose F. Vico Guzmán, Uwe Mittag, Sarah Michely, Edwin Mulder, Hirofumi Tanaka, Jens Tank, Jörn Rittweger

**Affiliations:** ^1^Facultad de Medicina, Instituto de Investigación Biomédica de Málaga, Universidad de Málaga, Málaga, Spain; ^2^German Aerospace Center (DLR), Institute of Aerospace Medicine, Cologne, Germany; ^3^College of Kinesiology, University of Saskatchewan, Saskatoon, SK, Canada; ^4^Department of Kinesiology and Health Education, The University of Texas at Austin, Austin, TX, United States; ^5^Department of Pediatrics and Adolescent Medicine, University of Cologne, Cologne, Germany

**Keywords:** aging, veteran athletes, anaerobic power, bio-impedance, phase angle, muscle, mechanography

## Abstract

Vertical jumping power declines with advancing age, which is theoretically explicable by loss of muscle mass and increases in body fat. However, the results of previous cross-sectional studies remain inconsistent on these relationships. The present study included 256 masters athletes who competed at the 2018 track and field world championships in Málaga, Spain. We assessed body composition with bioelectrical impedance (Inbody S10) and vertical jumping power with a Leonardo ground reaction force platform. Relationships between age, jumping power, and body composition were analyzed by correlation and regression analyses. Hierarchical multiple regression analysis was used to evaluate effects of each factor on vertical jumping power. Age-related rates of decreases in maximal power and jump height were similar between male and female athletes. Percent fat-free mass and percent body fat were negatively and positively, respectively, associated with age in masters athletes and were comparable to those previously observed in the general population. Moreover, these effects in body composition can, to a great extent, explain the age-related decline in jumping power, an effect that seems at least partly independent of age. Finally, the multiple regression model to determine independent predictors of vertical jump performance yielded an overall *R*^2^ value of 0.75 with the inclusion of (1) athletic specialization in power events, (2) percent fat-free mass, and (3) phase angle. However, partial regression yielded significant effects of age, but not gender, on peak power, even when adjusting for athletic specialization, percent fat-free mass, and phase angle. We concluded that loss of skeletal muscle mass and changes in bio-impedance phase angle are important contributors to the age-related reduction in anaerobic power, even in adults who maintain high levels of physical activity into old age. However, age per se remains a significant predictor of vertical jump performance, further demonstrating deteriorated muscle quality at old age (sarcosthenia).

## Introduction

Age-related physiological variations of body composition encompass both fat-free mass (FFM), which includes minerals (bone mass), proteins (muscle mass) and total body water, and fat mass (FM) (Wang et al., 2020). Dependent on the type of sport, athletic retirement is often characterized by a reduction in physical training stimuli causing loss of lean body mass and fitness as well as altered body composition (Liu et al., 2008). With the advancement of age, there is generally an increase in trunk fat (visceral fat) and a decrease in subcutaneous fat (Yarizadeh et al., 2020). Another characteristic related to old age is the accumulation of fat in non-fatty tissues (termed “ectopic” fat). Alterations in ectopic fat have been studied mainly in older adults, suggesting that the amount of intermuscular adipose tissue increases with age. Although age-related accumulation in intermuscular adipose tissue may be more visible in those with greater total body weight, it has also been observed in people with low body weight (Rossi et al., 2011). In addition, there is also an age-related accumulation of intra-muscular adipose tissue, and likely even in the intracellular lipid content, which is thought to hamper muscle’s mechanical functioning (Goodpaster et al., 2001; Correa-de-Araujo et al., 2020).

Age-related loss of muscle mass is referred to as sarcopenia (Visser, 2009; Narici and Maffulli, 2010), and the accompanying loss of function is referred to as dynapenia (Manini and Clark, 2012). Enhanced body fat and loss of muscle mass with age together increase the risks of developing sarcopenic obesity, characterized by the redistribution of subcutaneous fat and an excess of visceral adiposity associated with a reduction in muscle mass and strength (Stenholm et al., 2008; Zamboni et al., 2008; Dawson and Dennison, 2016). In a physical analogy to vehicles, one could equate the engine to the body’s musculature, and the vehicle’s load to excess adipose tissue. Reductions in the size (∼sarcopenia) and power (∼dynapenia) of the engine will slow down the vehicle, and this will be further aggravated by increasing the passive load (∼obesity). It is therefore no surprise that sarcopenia and dynapenia are associated with reduced vertical jump performance (Siglinsky et al., 2015) and reduced gait speed at old age (Studenski et al., 2011). Sarcopenia, dynapenia, and slow gait speed, in turn, are important predictors of dysmobility, loss of autonomy and death (Newman et al., 2006; Stanaway et al., 2011; Cruz-Jentoft, 2013). In addition to dynapenia, the term sarcosthenia has been proposed to describe poor quality of muscle tissue, which likely also contributes to the age-related decline in physical functioning (Tanaka et al., 2019).

Skeletal muscle retains a remarkable plasticity to be responsive to exercise training into very old age (Fiatarone et al., 1994). However, the readiness to exert oneself in exhaustive training sessions is often dwindling in the senior population. In this respect, masters athletes are an intriguing population, as they are driven by the desire to win the competitions that they participate in. They hitherto adhere to demanding training regimens in order to get their physique into the best possible shape. From a physiological point of view, they can accordingly be seen as a model of highly active aging (Rittweger et al., 2004a; Tanaka et al., 2019).

Over the past decades, the vertical jump test has been established as an intuitive test that has good ecological validity (Hong et al., 2020) and that depicts virtually no learning effect (Rittweger et al., 2004b). Another advantage above other physical tests like the chair rising test is that it is discriminative over a very wide spectrum of physical capability, ranging from elite athletes to frail patients (Hardcastle et al., 2014). In an initial cross-sectional study (Runge et al., 2004), normative data were generated to assess the age-related declines in peak neuromuscular power. This test calculates the peak power that is developed during a counter-movement jump and evaluates the entire chain of anti-gravity muscles required for many normal physiological activities. We have been using the vertical jump test in track and field masters athletes and found that the age-trend in sprinters and distance runners follow a trajectory that was parallel above and below the EFI-line, respectively (Grassi et al., 1991; Michaelis et al., 2008). Moreover, novel, longitudinal data confirm that individual athletes undergo an age-related decline in neuromuscular power that is well-predicted by the EFI score (A. Ireland, J. Rittweger et al., submitted).

The question is therefore arising whether the age-related decline in vertical jump power is due to sarcopenia (=muscle wasting), to sarcosthenia (=poor muscle quality), and/or to excess passive load (=obesity) in the masters athletic population. Addressing this question will help to better understand in how far deterioration in physical performance at old age is attributable to changes in body composition. Practically, this can improve our ability to predict performance via body composition assessments. So far, only sporadic and non-systematic studies exist on body composition in masters athletes (Tanaka et al., 2019), but modern bio-impedance analysis (BIA) can be used to assess body composition from the electrical properties of body tissue (Kyle et al., 2004). Multi-frequency approaches in particular can accurately estimate total body water (TBW), fat mass (FM), and fat-free mass (FFM), with the latter being highly correlated to muscle mass. The use of the bicompartmental model (2C) is therefore widespread in clinical practice and epidemiology. The overall aim of the present study therefore was to investigate whether age-related effects in body composition can explain the age-related decline in vertical jumping performance in masters athletes. Our working hypothesis was that decreases in vertical jump performance with advancing age can be explained largely by the corresponding changes in body composition in masters athletes, and that apparent age-effects would be explained in men and women alike across the range of different athletic specializations.

## Materials and Methods

The Masters Athletic Field Study 2018 (MAFS-18) aimed to assess physiological and mental constituents of fitness and well-being in masters athletes. It was implemented during the 23rd World Masters Athletics Championships held in Málaga, Spain between 4th and 15th September 2018, where 8,189 athletes registered for competitions. Data collection took place in the Málaga City Stadium in close proximity to the registration office. The study was approved by the Masters Athletics organizing committee, and the research protocol was reviewed and approved by the ethical commission of the North Rhine Medical Association (Ärztekammer Nordrhein lfd Nr 2018171). The study was registered with the German register for clinical trials^1^ with identifier DRKS00015172 before the commencement of the study. The only inclusion criterion was that participants competed in the championships. Injuries that interfered with the testing procedures were criteria for exclusion.

### Participants

Initially, the MAFS-18 study had been designed with a sample size of 60 to 120 participants. However, overwhelming interest on the side of the athletes allowed us to include a total of 256 masters athletes. Of these, 240 athletes aged between 35 and 91 years (mean 58 ± 12 years) participated in the present sub-study. All the participants provided their written informed consents.

### Study Flow

#### Basic Assessment

After inclusion, a brief questionnaire-guided interview was performed with the participants to assess information on athletic specialization, training habits, and medical conditions. Participants were also identified by their bib number, which was invariant throughout the Málaga competitions, and all participants consented for their personal data to be stored for future longitudinal analyses. Next, height and weight were assessed using a stadiometer (Kern MPE250 K100HM, Balingen, Germany) to the nearest of 0.1 cm and 100 g, respectively.

#### Vertical Jump Test

The test was performed with a Leonardo ground reaction force platform (Novotec Medical, Pforzheim, Germany) with the integrated software in its version 4.4b01.35 (research addition). This software screens the ground reaction force signal for a period in which movement-related variation is reduced below a critical threshold, to then provide a starting signal to participants. Stability of the force signal prior to the jump is essential, as accurate estimation of body mass *m* is required for the mathematical integrations from force *F* to velocity (∫ F/m) and to speed (∬ F/m) (Davies and Rennie, 1968; Rittweger et al., 2007). Power is then computed as the product of force and velocity, and the peak jump power is the greatest power observed during the push phase, normalized to body mass. Peak power is then normalized by the published reference data to yield the “Esslinger” fitness index (EFI), for which a value of 100% indicates an average age-adjusted result (Ward et al., 2009). Meanwhile, the validity of the EFI has been confirmed in several studies that included North-American, Korean and Japanese cohorts (Tsubaki et al., 2009; Hong et al., 2020). In addition to peak power and the EFI, the Leonardo software also automatically computes the height of the jump (Hmax) and the depth of the countermovement (Hmin). It is important to notice that Hmax is dependent on Hmin, but that peak jump power and EFI are not (Salles et al., 2011).

Participants commenced the test with a few warm-up jumps, after which they were asked to perform three maximal vertical jumps, with the instruction to raise the body as high as possible in the air. Subjects were given 30 to 90 s between jumps according to their own preference. Arms were allowed to swing freely, as long as no exaggerated movements were performed that could lead to an unnatural increase of jump height. After each jump, the validity of the result was ascertained on basis of the displacement curve being back to 0, and jumps were rejected if this criterion was not fulfilled. All jump tests were performed by the same investigator (E.M.) throughout the study.

#### Body Composition

All participants were subjected to Bioelectrical Impedance Analyzer (Inbody S10, South Korea) with a segmental multi-frequency approach (1 kHz, 5 kHz, 50 kHz, 250 kHz, 500 kHz, and 1 MHz), following the manufacturer’s guidelines, and also following recommendations for clinical application of bioelectrical impedance analysis (Kyle et al., 2004). All participants were asked not to take any foods or drinks and to avoid strenuous activity within 4 h before the testing. All parameters of BIA testing were obtained after removal of any metal parts from the body, and using a standard montage of outer and inner electrodes on the right hand and foot while patients lay down during 10 min before measurement with legs apart. Whole-body resistance (R) and reactance (Xc) were obtained by BIA using a single frequency, phase-sensitive 50 kHz. From the physical measurement, the integrated Inbody software computes body composition indicators including skeletal muscle mass (SMM), percent skeletal muscle mass (PSSM), soft lean mass (SLM), percentage of body fat (PBF), fat free mass (FFM), fat mass (FM), percent FFM (PFFM), percent FM (PFM), intracellular water (ICW), extracellular water (ECW), total body water (TBW), mineral content, and protein content. Phase angle was calculated using the following equation: phase angle (°) = arctan (reactance/resistance) × (180/π). Phase angle has been proposed as an indicator of body cell mass and integrity (Barbosa-Silva and Barros, 2005). Short-term precision (calculated as the coefficient of variation) on repeated R and Xc was 0.31% and 0.77%, respectively. BIA measurements were used to assess muscle mass. Using resistance and reactance measured by BIA, apendicular skeletal muscle mass (ASMM) was estimated using the Sergi’s equation (Sergi et al., 2015). Appendicular muscle mass index (ASMI, kg/m^2^) was calculated by dividing ASMM by height in squared meter.

### Data Management

Basic assessment data were collected with a customized Redcap data base (Harris et al., 2009, 2019). All personal identifiable data were exclusively stored on a separate safe server, together with a unique MAFS-18 pseudonymized identifier. These pseudonymized identifiers were used within the Leonardo (jump test) and Inbody (BIA) data bases, and data from the Redcap, Leonardo and BIA data bases were merged with customized R-scripts^2^.

From the 3 jumps performed by each athlete, we selected the jump with greatest height for further analysis. Athletic specializations were grouped into power, mixed, and endurance events, based on subjective rating of the best event by each athlete. Thus, there was only one data set for all variables per participant.

### Statistical Analyses

Normality was analyzed using the Kolmogorov-Smirnov test. Asociations between variables were assessed using Spearman’s rank correlation coefficients. For all correlation analyses, residuals were examined with residual plots and quantile-quantile plots in order to check for linearity of the relationship. This can be confirmed for all correlation results reported here. The following criteria were adopted to interpret the magnitude of the correlations: *r* < 0.1, trivial; 0.1 < *r* ≤ 0.3, small; 0.3 < *r* ≤ 0.5, moderate; 0.5 < *r* ≤ 0.7, large; 0.7 < *r* ≤ 0.9, very large; and *r* > 0.9, almost perfect (Hinkle et al., 2003).

Mann Withney *U* test were performed for comparisons between sexes. A one-way ANOVA with post hoc of Student-Newman–Keul or Kruskall-Wallis test with post hoc of Conover, when appropriate were applied to test differences between athletic specializations (Power = sprinters, throwers and jumpers; Mixed = middle-distance, combined events, and Endurance = 5,000 m, 10,000 m, road walk, and marathon). Variables significantly associated with jump test performance (independent variables) were included in a stepwise multiple regression analysis to estimate the predictors of jump performance test (dependent variables). These variables were selected because they did not violate the collinearity diagnosis (variance inflation factor < 10 and tolerance > 0.2) (Kutner et al., 2004).

Descriptive and correlation statistical analyses were carried out with the MedCalc statistical software, version 19.4.0 (Ostend, Belgium). The data are presented as medians and 95% confidence intervals (CI). Multiple regression analyses were also replicated with the “lm” command within the R-software (see text footnote 2), and partial *R*^2^-values were assessed with the function “r2beta” of the R-package “r2glmm.” A *P* < 0.05 was considered for statistical significance. Finally, partial correlation analyses were performed with the R-software, in order to establish whether residuals of the regression between jump performance variables (peak power, EFI, Hmax and Hmin = dependent variables) and athletic specialization, PFFM, and phase angle (= independent variables) were correlated with age and sex.

## Results

### Sex Differences in Body Composition and Jump Test Performance

Anthropometric measures, body composition, and vertical jump test performance of male and female masters athletes can be seen in Table 1. As expected, males were heavier and taller than females (*P* < 0.001). All body composition variables, except fat mass (*P* = 0.67), have higher values in males compared with females (*P* < 0.0001). All the variables derived from the vertical jump test were greater in male than in female masters athletes (all *P* < 0.05).

**TABLE 1:** Comparisons of body composition and vertical jump performance between male and female masters athletes.

**Variables**	**Male (*n* = 162)**		**Female (*n* = 91)**		***P*-value**
	**Median**	**95% CI**	**Median**	**95% CI**	
Age (years)	58.0	56.0−61.0	55	52.0−57.3	0.058
Weight (kg)	72.6	71.6−74.0	59	57.7−62.2	<0.0001
Height (cm)	173.9	172.3−174.8	164.1	162.0−165.1	<0.0001
BMI (kg/m^2^)	24.4	24.0−24.8	22.5	21.4−23.4	<0.0001
BFM (kg)	13.4	12.2−14.5	12.6	11.3−14.8	0.672
PBF (%)	18.4	17.5−20.1	21.1	19.8−24.4	<0.0001
FFM (kg)	59.4	57.1−60.8	45.6	44.5−48.0	<0.0001
FFM (%)	81.4	79.8−82.5	78.8	75.8−80.1	<0.0001
TBW (%)	43.5	42.0−44.7	33.5	32.5−35.2	<0.0001
TBW (kg)	59.8	58.5−60.5	57.4	54.9−58.5	<0.0001
ICW (%)	27.1	57.1−60.8	20.6	21.0−21.7	<0.0001
ICW (kg)	37.0	57.1−60.8	35.3	34.4−36.1	<0.0001
ECW (%)	16.4	15.9−17.2	12.9	12.4−13.5	<0.0001
ECW (kg)	22.7	22.3−23.1	22.0	21.1−22.3	0.0001
WB resistance (Ω)	516.3	478.0−564.1	587.1	538.7−630.3	<0.001
WB reactance (Ω)	56.2	52.0−62.9	60.1	54.1−66.6	0.07
WB impedance (Ω)	519.2	480.6−566.7	590.6	542.8−633.1	<0.001
WB PhA (°)	6.3	6.1−6.4	5.7	5.6−5.9	<0.0001
ASM/Height^2^ (kg/m^2^)	7.05	6.6−7.4	5.9	5.6−6.4	<0.001
ASMM (kg)	20.9	19.3−23.2	1.2	14.6−18.2	<0.001
EFI	96.0	92.5−99.0	98.6	95.8−106.2	0.019
EFIzScore	–0.24	−0.451-−0.05	–0.08	−0.25−0.4	0.015
Peak power (W/kg)	38.8	36.040−40.5	32.91	29.5−35.2	<0.0001
Peak Accel (W/kg)	2.2	2.164−2.2	2.06	2.0−2.1	0.002
H max CMJ (m)	0.35	0.340−0.37	0.29	0.26−0.30	<0.0001
Hmin CMJ (m)	–0.29	−0.31−0.28	–0.25	−0.27−0. 20	<0.0001

*BMI, body mass index; BFM, body fat mass; PBF, percent body fat; FFM, fat-free mass; TBW, total body water; ICW, intracellular water; ECW, extracellular water; ASM, appendicular skeletal muscle; ASMM, appendicular skeletal muscle mass; WB, whole body; PhA, phase angle; EFI, Esslingen fitness index; CMJ, countermovement jump; H_max_CMJ, jump height in CMJ; H_min_CMJ, countermovement depth in CMJ.*

### Body Composition and Jump Test Performance Among Athletes With Different Athletic Specialization

Age, percentage of body composition variables, including body fat, soft lean mass, fat-free mass, and skeletal muscle mass were not different between sport disciplines (all, *P* > 0.05). Body composition variables expressed in kg (FFM, SLM) were significantly different between the groups (see pairwise comparisons in Table 2), (all *P* < 0.0001). Most vertical jump test performance variables except for Hmin were significantly different between the athletic groups (*P* < 0.001).

**TABLE 2:** Body composition and vertical jump performance of athletes in different athletic specialties.

**Variables**	**Power (*n* = 135)**		**Mixed (*n* = 40)**		**Endurance (*n* = 69)**		***p***	**PC**
	**Median**	**IQR**	**Median**	**IQR**	**Median**	**IQR**		
Age (years)	56.0	47.0−65.0	65.0	52.5−71.0	57.0	50.0−64.2	0.064	
Weight (kg)	71.7	66.3−79.1	67.0	58.5−75.4	63.5	57.3−72.0	<0.001	a.b
Height (cm)	171.9	166.0−177.2	170.2	165.2−178.2	167.2	161.2−172.0	0.001	b.c
BMI (kg/m^2^)	24.5	22.8−25.9	22.6	20.6−25.1	22.9	21.2−24.6	0.001	b
BFM (kg)	27.2	19.3−35.6	27.5	22.3−36.0	32.0	25.1−39.5	0.54	
PBF (%)	20.0	14.3−25.5	18.2	14.7−21.0	20.1	16.8−25.8	0.65	
FFM (kg)	57.5	49.9−64.9	53.6	48.0−58.5	50.5	45.0−56.3	<0.001	b.c
FFM (%)	79.9	74.5−85.6	81.7	77.0−85.3	79.9	74.2−83.1	0.64	
TBW (%)	42.2	36.8−47.7	39.3	35.3−42.9	37.3	33.1−41.2	<0.001	b
ECW (%)	15.9	14.2−17.9	15.0	13.6−16.7	14.2	12.7−15.8	<0.001	b.c
ICW (%)	26.3	22.7−29.7	24.4	21.5−26.6	22.9	20.1−25.5	<0.001	a.b
WB resistance (Ω)	526.1	478.7−584.8	561.4	509.0−606.7	559.8	513.7−598.5	0.012	b
WB reactance (Ω)	57.0	52.9−63.2	57.5	50.1−65.2	58.8	53.1−65.5	0.66	
WB impedance (Ω)	527.6	482.4−587.6	564.4	513.3−610.9	563.0	516.6−602.2	0.013	b
WB_PhA (°)	6.3	5.7−6.9	5.8	5.4−6.3	5.7	5.3−6.2	<0.001	a.b
ASM/Height^2^ (kg/m2)	6.9	6.2−7.3	6.5	5.7−7.0	6.7	5.9−7.0	0.011	a. b
ASMM (kg)	20.4	17.5−22.9	18.7	15.1−20.7	19.1	16.2−21.1	0.017	b
EFI	105.6	94.9−119.1	95.7	87.2−107.1	83.8	73.0−92.5	<0.001	a.b.c
EFIzScore	0.3	−0.3−1.1	–0.2	−0.7−0.4	–0.9	−1.6−0.4	<0.001	a.b.c
Peak power (g)	41.4	35.0−47.4	34.2	29.6−38.9	30.7	27.8−33.7	<0.001	a.b.c
Peak accel (g)	2.2	2.0−2.5	2.1	2.0−2.3	2.0	1.8−2.2	<0.001	a.b
H max CMJ (cm)	0.3	0.3−0.4	0.3	0.2−0.3	0.2	0.2−0.3	<0.001	a.b
H min CMJ (cm)	–0.2	−0.3−0.2	–0.2	−0.3 to −0.2	–0.2	−0.3−0.2	0.58	

*BMI, body mass index; BFM, body fat mass; PBF, percent body fat; FFM, fat-free mass; PFFM, percent Fat-free mass; TBW, total body water; ICW, intracellular water; ECW, extracellular water; ASM, appendicular skeletal muscle; ASMM, appendicular skeletal muscle mass; WB, whole body; PhA, phase angle; EFI, Esslingen fitness index; CMJ, countermovement jump; H_max_CMJ, jump height in CMJ; H_min_CMJ, countermovement depth in CMJ; PC, pairwise comparisons (a, diff power vs. mixed; b, diff power vs. endurance; c, diff mixed vs. endurance).*

### Age-Related Changes in Vertical Jump Performance

The age-related rates of declines in maximum power and Hmax in vertical jump performance were similar in both male and female athletes as evidenced by similar slopes (Figure 1). When masters athletes were divided into different athletic specialties, power and mixed athletes demonstrated greater decreases in vertical jump performance than endurance athletes. The age-associated decreases in peak acceleration were similar between sexes but were statistically greater in the Power group. Age-related effects in Hmin were similar between sexes (equal slopes); these effects were significant in the power and mixed groups (Tables 3A,B).

**FIGURE 1:** Age dependency of vertical jump test performance of Master Athletes. At left: Comparison of variables by gender. At right: Comparisons of variables by sport specialty. Regression lines and equations are represented and consigned when they are significant (see correlation coefficients between variables in Tables 3A,B).

**TABLE 3:** **(A)** Spearman’s rank correlation coefficients between age and vertical jump performance stratified by sex. **(B)** Spearman’s rank correlation coefficients between age and vertical jump performance stratified by athletic specialty.

**(A)**							
**Variable**	**Group**	***n***	**Peak power CMJ**	**Peak Acc CMJ**	**H max CMJ**	**H min CMJ**	**EFI**
Age	All	238	−0.53***	−0.25***	−0.56***	0.34***	0.13*
	Male	153	−0.59***	−0.29**	−0.66***	0.39***	0.27**
	Female	85	−0.68***	−0.29***	−0.69***	0.44***	–0.08

**(B)**							
	**Group**	***n***	**Peak power CMJ**	**Peak Acc CMJ**	**H max CMJ**	**H min CMJ**	**EFI**

Age	Power	131	−0.65***	−0.27*	−0.66***	0.35***	0.08
	Mixed	36	−0.59**	–0.28	−0.62***	0.41*	0.41*
	Endurance	65	−0.43**	–0.24	−0.43**	0.21	0.30*

Acc, acceleration; CMJ, countermovement jump; H, height; EFI, Esslingen fitness index. *P < 0.05, **P < 0.001, ***P < 0.0001.

### Age-Related Changes in Body Composition

Body composition variables including body weight, PSLM, PFFM (all, small correlations) and whole-body phase angle (moderate correlation) were inversely and percent body fat was directly correlated with age (Figure 2). The highest correlation with age was observed with phase angle (*r* = 0.42 to 0.69, all *P* < 0.001) as shown in Tables 4A,B. Body weight tended to decrease with increasing age in the group of males but not in females. There was no difference in age-related changes in body weight among different athletic groups (*P* < 0.05).

**FIGURE 2:** Age dependency of body composition variables of Master Athletes. At left: Comparison of variables by gender. At right: Comparisons of variables by sport specialty, WB PhA, whole body phase angle, regression lines, and equations are represented and consigned when they are significant (see correlation coefficients in Tables 4A,B).

**TABLE 4:** **(A)** Spearman’s rank correlation coefficients between age and body composition stratified by sex. **(B)** Spearman’s rank correlation coefficients between age and body composition stratified.

**(A)**								
**Variable**	**Group**	***n***	**Weight**	**PBF**	**PSLM**	**PFFM**	**PSMM**	**WB PhA**
Age	All	252	–0.03	0.29***	−0.28***	−0.29***	−0.34***	−0.59***
	Male	161	−0.18*	0.36***	−0.35***	−0.35***	−0.45***	−0.68***
	Female	91	–0.04	0.28*	−0.27*	−0.28*	−0.37**	−0.65***

**(B)**								
Age	Power	134	–0.10	0.38***	−0.38***	−0.39***	−0.44***	−0.69***
	Mixed	40	0.10	0.14	–0.13	–0.14	–0.25	−0.48*
	Endurance	65	0.06	0.06	–0.05	–0.06	–0.15	−0.43**

PBF, percent body fat; PSLM, percent soft lean mass; PFFM, percent fat-free mass; PSMM, percent skeletal muscle mass; WB PhA, phase angle whole body. *P <0.05, **P < 0.001, ***P < 0.0001.

### Relations Between Body Composition and Vertical Jump Performance

Percent body fat was inversely correlated with vertical jump performance (*r* = −0.13 to −0.55, all *P* < 0.05) except Hmin that had direct correlation. In general, greater degrees of correlations were seen in female athletes than in male athletes (Table 5 and Figure 3).

**TABLE 5:** Spearman’s rank correlation coefficients between percent body fat and phase angle with vertical jump performance in male and female athletes.

**Variable**	**Group**	***n***	**Peak power CMJ**	**Peak Acc CMJ**	**H max CMJ**	**H min CMJ**	**EFI**
PBF	Male	150	−0.36***	−0.21*	−0.45***	0.24*	−0.14*
	Female	83	−0.55***	−0.36**	−0.49***	0.41***	−0.45***
WB PhA	Male	150	0.67***	0.37***	0.67***	−0.32***	0.10
	Female	83	0.81***	0.26*	0.83***	−0.47***	0.44***

Acc, acceleration; CMJ, countermovement jump; H, height; EFI, Esslingen fitness index; PBF, percent body fat; WB PhA, whole body phase angle. *P < 0.05, **P < 0.001, ***P < 0.0001.

**FIGURE 3:** Body composition dependency of vertical jump test variables of master athletes. At left, percent body fat dependency of vertical jump test variables. Comparison of variables by gender. At right, Phase angle dependency of vertical jump test variables. Comparisons of variables by gender, WB PhA, whole body phase angle, regression lines, and equations are represented and consigned when they are significant (see correlation coefficients in Table 5).

### Relation Between Phase Angle and Vertical Jump Performance

Phase angle presented moderate correlations in males (*r* = −0.32 to 0.67, *P* < 0.0001) and larger correlation coefficients in females (*r* = −0.47 to 0.82, *P* < 0.0001) with vertical jump performance variables. Esslingen fitness Index (EFI) was correlated with phase angle in females but not in males (Table 5 and Figure 3).

### Independent Determinants of Vertical Jump Performance

Table 6 features the multiple linear regression analyses showing independent predictor variables for vertical jump performance, including age, sex, athletic group, and body composition variables (stepwise method). Seventy five percent of the variance (*P* < 0.001) in peak power was explained by age, athletic group, sex, PFFM and whole body phase angle. The same independent variables plus BMI were predictors of Hmax (*R*^2^ = 0.75, *P* < 0.001). Coefficients of determination for peak acceleration (*R*^2^ = 0.23, *P* < 0.001) and Hmin (*R*^2^ = 0.31, *P* < 0.001) were small to moderate, and for EFI (*R*^2^ = 0.55, *P* < 0.001) large.

**TABLE 6:** Multiple regression analyses to predict independent determinants of vertical jump performance.

**Models**	***n***	***R*^2^**	***R*^2^-adj.**	**MCC**	**RSD**	
Peak power (W/kg)	227	0.75	0.75	0.87	4.60	
Peak Accel (g)	226	0.23	0.22	0.48	0.26	
H max CMJ (cm)	226	0.75	0.75	0.87	48.5	
H min CMJ (cm)	227	0.26	0.25	0.56	0.06	
EFI (%)	226	0.55	0.54	0.74	12.44	

**(A) Regression equation to predict peak power (W/kg)**						
**Independent variables**	**Coefficient**	**Std. error**	***T***	***P***	**VIF**	**Partial *R*^2^**

Constant (W/kg)	12.74	6.86	1.86	0.065		
AthGr	−4.022	0.372	−10.81	<0.0001	1.11	0.35
PFFM (%)	0.282	0.047	5.94	<0.0001	1.63	0.14
WB_PhA (°)	4.008	0.605	6.63	<0.0001	2.55	0.17
Age (years)	−0.201	0.036	−5.64	<0.0001	2.01	0.13
Sex	−2.893	0.762	−3.80	0.00019	1.48	0.06

**(B) Regression equation to predict peak acceleration (g)**						
**Independent variables**	**Coefficient**	**Std. error**	***T***	***P***	**VIF**	**Partial *R*^2^**

Constant (g)	1.063	0.205	5.18	<0.0001		
WB_PhA	0.093	0.026	3.625	0.0004	1.33	0.06
AthGr	−0.075	0.021	−3.61	0.0004	1.07	0.06
PFFM	0.0088	0.0026	3.329	0.0010	1.25	0.05

**(C) Regression equation to predict Hmax CMJ (cm)**						
**Independent variables**	**Coefficient**	**Std. error**	***T***	***P***	**VIF**	**Partial *R*^2^**

Constant (cm)	−14.37	11.72	−1.23	0.22		
AthGr	−3.06	0.405	−7.12	<0.0001	1.19	0.21
Age (years)	−0.271	0.038	−7.55	<0.0001	2.02	0.19
PFFM (%)	0.515	0.086	5.98	<0.0001	4.20	0.14
BMI (kg/m^2^)	0.684	0.196	3.49	0.0006	2.87	0.05
Sex	−3.144	0.900	−3.45	0.0006	1.90	0.05
WB_PhA (°)	2.642	0.708	23.73	0.0002	3.31	0.06

**(D) Regression Equation to predict Hmin CMJ (cm)**						
**Independent variables**	**Coefficient**	**Std. error**	***T***	***P***	**VIF**	**Partial*R*^2^**

Constant (cm)	−2.20	7.35	−0.30	0.76		
PSLM	0.284	0.072	−3.98	<0.0001	1.29	0.07
Age	0.134	0.046	289	0.0043	1.57	0.04
WB_PhA	−1.86	0.77	−2.42	0.016	1.80	0.02

**(E) Regression equation to predict EFI (%)**						
**Independent variables**	**Coefficient**	**Std. error**	***T***	***P***	**VIF**	**Partial *R*^2^**

Constant (%)	−65.7	18.6	−3.53	0.0005		
AthGr	−10.6	1.01	−10.6	<0.0001	1.11	0.34
Sex	18.3	2.06	8.88	<0.0001	1.47	0.26
Age (years)	0.747	0.096	8.03	<0.0001	2.01	0.23
PFFM (%)	0.814	0.128	6.34	<0.0001	1.62	0.16
WB_PhA (°)	7.983	1.639	4.87	<0.0001	2.41	0.10

*Accel, acceleration; AthGr, athletic group (1, power; 2, mixed; and 3, endurance); EFI, Esslingen fitness index; Hmin, depth of the countermovement; Hmax, jump height; MCC, multiple correlation coefficient; PFFM, percent fat-free mass; PFMM, percent fat-free mass; PSLM, percent soft lean mass; *R*^2^, coefficient of determination; *R*^2^- adj, *R*^2^ adjusted; RSD, residual standard deviation; Sex, 0 for female and 1 for male; VIF, variance inflation factor; WB_PhA, whole body phase angle.*

Partial correlation analyses yielded a significant correlation of the residuals of the model *peak power = athletic specialization + PFFM + phase angle + error* were significantly correlated with age (*P* < 0.001), but not with sex (*P* = 0.08), suggesting that body composition and athletic specialization fully explain sex effects but not age effects in the current peak power data set. For Hmax, by contrast, both age (*P* < 0.001) and sex (*P* = 0.005) were correlated with residuals, and Hmin also showed weakly significant partial correlations for age (*P* = 0.018) and sex (*P* = 0.12) (Table 6).

Finally, looking at the relationship between fat-free mass and the predicted skeletal mass, correlation coefficients of 0.9985 and of 0.985 were found (both *P* < 0.001) for SMM vs. FFM and for PSSM *vs*. PFFM, respectively. According to the obtained regression coefficients, SMM was linked to −2.8 kg + 0.607 ^∗^ FFM, and PSSM was linked to −4.3% + 0.610 ^∗^ PFFM in the present data.

## Discussion

The present study has demonstrated the expected relationship of age and sex on peak vertical jump power, which had previously been demonstrated in a non-athletic cohort (Siglinsky et al., 2015) aged 27–96 years, as well as in an masters athletes (Michaelis et al., 2008). In addition, we provided novel data on body composition in competitive masters athletes. Although previous studies on this topic had either used technology that is no longer state-of-the art (Grassi et al., 1991) or had included much smaller study samples than the present study (Pollock et al., 1987, 1997; Korhonen et al., 2003), these previous studies are in agreement with the present results that the relative fat content increases with increasing age even in competitive masters athletes. Thus, the present data suggest an age-related exaggeration in body fat percentage by 2.0 % (SE 0.4%) per decade, a change that is in remarkably good agreement with a previous longitudinal study in masters distance runners (Pollock et al., 1997). Notably, subjects were generally well hydrated (Table 1).

The question arises in which organs and compartments of the masters athletes it is that these lipids accumulate over time. From the physical appearance of most masters athletes, one does not have the impression that this accumulation would be occurring in the subcutaneous or abdominal adipose tissue. Previous studies in which we used peripheral quantitative computed tomography in masters athletes likewise did not reveal eye-striking expansion of subcutaneous adipose tissue in the leg or forearm at old age (Wilks et al., 2009). We therefore favor the explanation by age-related myosteatosis, which is nowadays a well-established phenomenon at old age (Miljkovic and Zmuda, 2010), and which seems to be related to unfavorable metabolic alterations (Zoico et al., 2013).

Of all the variables derived from BIA, it was notably the 50kHz phase angle that depicted the greatest correlation with age. This resonates with a previous study that found phase angle and muscle cell mass were significant predictors of vertical jump performance in a non-athletic cohort aged 26–76 years (Yamada et al., 2017). Generally, the use of BIA has gained momentum in nutritional studies, and phase angle is a direct measure of BIA that is not influenced by algorithmic computations to assess body composition compartments (Bosy Westphal et al., 2006). Phase angle is thus a robust variable of its own interest in BIA because it is not dependent on height and weight. In addition, these measurements are related to cell membrane function, and they are an indicator of tissue hydration and nutritional condition (Barbosa-Silva and Barros, 2005). Phase angle reflects the electrical property of the tissues, whereby low values are associated with reduced cell unity, and higher values are associated with active cell mass, indicating an adequate state of health (Selberg and Selberg, 2002). Phase angle variability is related to cell composition and function as well as the redistribution of fluids and their changes through the interstitial spaces (Baumgartner et al., 1988). Bioelectrical impedance-derived phase anngle has been used to assess cellular health in various populations, and also as a tool for predicting muscular performance in the general population and in adult athletes (Hetherington-Rauth et al., 2020). For BIA measurements, participants were placed in a supine position for 10 min. Participants were also instructed to be on a fast conditions and a rest period of 12 h. Phase angle (PhA), a raw parameter derived from bioelectric impedance analysis (BIA), has been used as a marker for cellular functioning and to determine people’s health status, with applications in many clinical populations (Bosy Westphal et al., 2006). PhA has been correlated with muscle mass (Basile et al., 2014) as well as its characteristics (Cunha et al., 2018). Moreover, phase angle predicts the intracellular water pool (Francisco et al., 2020), as well as muscle strength and power in young athletes (Francisco et al., 2020).

Turning to the main objective of this study, namely the inter-relationship between body composition and the age-related decline in vertical jump power, multiple regression analysis has confirmed the initial hypothesis that the age-related decline in jump power is partly explained by lack of muscle mass. This is evidenced by the fact that PFFM and whole-body phase angle had a partial *R*^2^-values of 0.14 and 0.17, respectively (see Table 6A). Thus, these two BIA-derived measures each contributed more determination to the model than age (partial *R*^2^ = 0.13). PFFM was highly correlated with PSSM in the present data, and this strongly suggests that sarcopenia and potentially also age-related lipid accumulation are important factors in dynapenia as assessed by peak jump power. The fact that age still retained a substantial partial *R*^2^ in that multiple regression suggests that sarcosthenia (i.e., age-related muscle properties) is an independent another causative factor. Finally, it is pointed out here that the greatest determination was exerted by athletic specialization (partial *R*^2^ = 0.34). This implies that athletes maintain their athletic predisposition, and that power athletes have greater jump power than mixed event or endurance athletes throughout their lifespan.

Results for jump height, the second most informative value from the vertical jump test, share many similarities with results for peak power, namely strong determination by athletic specialization, age, PFFM, sex, and phase angle. It needs to be considered, though, that jump height is strongly affected by the countermovement depth (Vanrenterghem et al., 2004; Salles et al., 2011), which was assessed as Hmin in this study, and did not vary greatly with age (partial *R*^2^ = 0.07). However, given that the algorithmic computation is more robust for power than for height, peak power seems a better choice as study endpoint than jump height.

Finally, it is interesting to see that unlike the other aforementioned studies (Tsubaki et al., 2009; Hong et al., 2020), EFI depicted an age-trend, albeit a moderate one. As can be seen in Figure 1, older age was associated with greater EFI-values. These obvious positive deviations from the age-related decline in neuromuscular power observed here may suggest that masters athletes benefit from some sparing effect through their continued and often life-long athletic participation. When applying the cut-off values, that were found by Hong et al. (2020) in an inter-cultural comparison in vertical jumping power (19 W/kg and 23.8 W/kg for women and men, respectively), and the cut-off values for appendicular skeletal muscle mass by bio-electrical impedance we found only one subject within our cohort of over 200 participants who fulfilled the criterion for sarcopenia (Cruz-Jentoft et al., 2010). This was race walker in his 8th decade of life with body mass index of 23.9 and 28% body fat.

### Limitations

The present study has been a field study, and it was thus impossible to use dual energy x-ray absorptiometry (DEXA) for estimation of lean mass. However, DEXA is associated with a risk of radiation exposure, and one cannot study women who are potentially pregnant. Moreover, the Inbody S10 machine used in the present study for bioelectrical impedance analysis hast demonstrated good validity against DEXA measurements in an elderly population. Thus, we argue that bio-impedance measurements are an acceptable compromise for a field study. One could also ask why there has been no “control” group in the study. However, the comparator in the present study has been the athletic group, as our specific interest was to study the contribution of body composition effects to physical performance decline in aging athletes. However, there were only 5 participants in the present study who were older than 80 years, and only 31 were older than 70 years, so that no conclusions can be drawn on the prevalence of sarcopenia in the masters athletes.

In conclusion, the present study has provided evidence from 240 highly trained track and field athletes to suggest that muscle loss and fat accumulation are occurring also in this population, as in the general population. Reduced muscle mass and accumulated fat both explain significant portions of the age-related decline in vertical jumping performance. However, age remained strongly significant in partial correlation analysis for peak power after adjustment for PFFM, phase angle and athletic specialization. The effects of sex, conversely, upon peak power were fully explained by body composition and athletic specialization, which enhances our trust in the present results. The present data are therefore compatible with sarcosthenia as an additional, age-related factor to account for dynapenia. Future studies should explore to which extent the combined assessment of vertical jump power and body composition can be used to assess an individual’s fitness, and whether the information obtained is predictive of hard clinical endpoints such as bad health, dysmobility, and death.

## Data Availability Statement

The raw data supporting the conclusions of this article will be made available by the authors, without undue reservation.

## Ethics Statement

The studies involving human participants were reviewed and approved by Ethical Committee of the North Rhine Medical Association (Ärztekammer Nordrhein lfd Nr 2018171). The study was registered with the German register for clinical trials (www.drks.de) with identifier DRKS00015172 before the commencement of the study. The patients/participants provided their written informed consent to participate in this study.

## Author Contributions

JR designed the experiment. MB, EM, JV, HT, PC, JA-C, SM, and PF-M recruited the subjects and performed the experiments. UM and JR processed the data. JA-C and JR analyzed the data and drafted the manuscript. JA-C, HT, PC, JT, and JR critical revision of the article for important intellectual content. All authors gave final approval of the version to be submitted.

## Conflict of Interest

The authors declare that the research was conducted in the absence of any commercial or financial relationships that could be construed as a potential conflict of interest.

## Footnotes

1 www.drks.de

2 www.r-project.org/
